# Cancer Classification with a Cost-Sensitive Naive Bayes Stacking Ensemble

**DOI:** 10.1155/2021/5556992

**Published:** 2021-04-26

**Authors:** Yueling Xiong, Mingquan Ye, Changrong Wu

**Affiliations:** ^1^School of Medical Information, Wannan Medical College, Wuhu 241002, China; ^2^School of Computer and Information, Anhui Normal University, Wuhu 241002, China

## Abstract

Ensemble learning combines multiple learners to perform combinatorial learning, which has advantages of good flexibility and higher generalization performance. To achieve higher quality cancer classification, in this study, the fast correlation-based feature selection (FCBF) method was used to preprocess the data to eliminate irrelevant and redundant features. Then, the classification was carried out in the stacking ensemble learner. A library for support vector machine (LIBSVM), *K*-nearest neighbor (KNN), decision tree C4.5 (C4.5), and random forest (RF) were used as the primary learners of the stacking ensemble. Given the imbalanced characteristics of cancer gene expression data, the embedding cost-sensitive naive Bayes was used as the metalearner of the stacking ensemble, which was represented as CSNB stacking. The proposed CSNB stacking method was applied to nine cancer datasets to further verify the classification performance of the model. Compared with other classification methods, such as single classifier algorithms and ensemble algorithms, the experimental results showed the effectiveness and robustness of the proposed method in processing different types of cancer data. This method may therefore help guide cancer diagnosis and research.

## 1. Introduction

Cancer is a malignant tumor originating from epithelial tissues. It is a disease caused by the loss of normal regulation and the excessive proliferation of cells in the body. In recent years, cancer incidence and mortality have increased, thus posing severe risks to human health and life. In addition, because the occurrence and development of cancer are dynamic, most patients are diagnosed with cancer in late stages, thus making clinical diagnosis and treatment challenging [1, 2]. With the continual development of DNA microarray technology, gene expression profile data are gathered by synchronously tracking the expression of many genes. Consequently, early physiological information on cancer can be determined at the molecular level, and the type of cancer can be identified and used to guide biomedicine. However, many features are irrelevant and redundant for classification in gene expression profiles. Moreover, massive computational challenges, such as high dimensionality, small sample sizes, high noise, and unbalanced categories, introduce difficulties in the analysis and processing of cancer gene data. Therefore, various powerful methods have been proposed by researchers to address these problems [3].

At present, the application of machine learning methods to cancer classification is a significant research field in bioinformatics [4, 5]. Many traditional machine learning methods have been successfully applied to the classification analysis of gene expression data [6–9], such as RF, decision tree, KNN, and neural networks. However, with the increasing amounts and diversification of data, the traditional classification algorithm has been unable to meet the requirements of processing existing data and solving practical problems [10, 11]. Ensemble learning is a notable research direction in machine learning, in which multiple base learners are used for combined learning, and the combined classifier is often more accurate than its base classifier, thereby improving performance in classification problems. Combined classification algorithms have consequently been widely applied in classification problems [12, 13].

Boosting [14] and bagging [15] are two popular combined classification methods. Among them, bagging is a typical representative of a parallel ensemble learning method [16]. In this method, new training subsets are generated by adopting random sampling with putting back on the training set; then, individual learners are trained with different training subsets, respectively, and finally, they are integrated as a whole [17]. In this sampling process, it is inevitable that some instances will be sampled multiple times while others will be ignored [18]. Therefore, for a specific subspace, the individual learner will have high classification accuracy, while for those neglected parts, the individual learner is difficult to correctly classify [19]. In addition, the classification performance of the bagging method depends on the stability of its base classifier. It has a good classification effect for unstable classification algorithms (such as decision tree, neural network, etc.), but it is not very ideal for stable classifier integration [20]. Different from bagging, boosting is an iterative algorithm that transforms weak learners into strong ones [21]. A new weak classifier is added to each round to produce a strong learner with superior performance by increasing the number of iterations. Although the algorithm improves the generalization performance of the combined classification algorithm, the algorithm will suffer from performance degradation and long training time due to the excessive tendency to some difficult samples and the fact that the update of each round of sample distribution depends on the accuracy of the previous round of classifiers [13, 19, 20].

Compared with the two ensemble classification algorithms of bagging and boosting, stacking [22] provides a novel idea for ensemble learning, by emphasizing the deviations of the classifier from the training set and then learning these deviations to enhance classification performance. Stacking improves flexibility in combining learners that provide category output. In addition, this algorithm uses multiple types of individual classifiers to form a two-layer combined classification model. The first layer adopts multiple base learners to train the datasets, and a metalearner is used in the second layer to learn the output of the base learners [16, 18]. Generally, to avoid the overfitting caused by directly using the training sets of the primary learner, cross-validation is usually used to generate the new secondary training set. In addition, how to choose the data type of the secondary training set and the best secondary learner are the two key points that the algorithm must solve [19]. In recent years, stacking ensemble learning methods have been successfully applied in many fields [21]. For example, Ekbal and Saha [23] proposed the extraction of biomedical entities with combined feature selection and a stacking ensemble. The feature selection technique based on genetic algorithms was used to determine the most relevant feature sets of the support vector machine and conditional random field classifiers. Kwon et al. [22] applied a stacking ensemble to breast cancer classification and achieved better classification performance by using a gradient boosting machine and generalized linear model as metaclassifiers. Wang et al. [24] proposed a decision tree ensemble method based on stacking for prostate cancer detection, which achieved good results in classification accuracy, sensitivity, and specificity.

To further explore the effects of ensemble learning applied to cancer gene expression data, we adopted a two-layer classification model using a stacking ensemble learning strategy in combination with feature selection technology to conduct a classification study on binary cancer datasets. First, the original gene expression dataset was standardized and transformed into data with a mean value of 0 and a standard deviation of 1. Then, we used FCBF to calculate the *C*-correlation value of each gene and category through symmetric uncertainty, and the irrelevant genes were eliminated. The *F*-correlation value between features was calculated to eliminate the redundant genes and obtain the candidate gene subset, so as to simplify the combined classification model. Second, in the multiclassifier combination method based on the stacking algorithm, LIBSVM, KNN, C4.5, and RF were used as primary learners. Given the problem of imbalanced cancer gene expression data, CSNB was used as the metalearner of the stacking ensemble to perform combinatorial learning, which was expressed as CSNB stacking. Nine cancer datasets were tested for experiments and then compared with other single classifier algorithms and ensemble algorithms: cost-sensitive KNN stacking (CSKNN stacking), cost-sensitive C4.5 stacking (CSC4.5 stacking), cost-sensitive LIBSVM stacking (CSLIBSVM stacking), bagging, AdaBoost, CSNB, NB, LIBSVM, KNN, RF, and C4.5. The experimental results demonstrated that the proposed method provided more accurate classification and was effective and robust in handling various cancer classification data.

The rest of the paper is organized as follows.  Section 2 reviews the related work about cancer classification problem.  Section 3 introduces the materials and methods of this study, and Section 4 exhibits and discusses the experimental results. In the end, we summarize the paper.

## 2. Related Work

The mature development of DNA microarray technology provides important guidance for cancer diagnosis and recognition. At present, many scholars have applied the machine learning method to cancer classification and thus designed various classification models and achieved satisfactory results. For example, Musheer et al. [25] used a naive Bayes classifier to classify and evaluate six microarray cancer datasets after feature reduction, which proved that the algorithm has certain significance. Ye et al. [1] applied the KNN classifier to evaluate the extracted information gene subset, which improved the classification accuracy. Besides these, there are also some classification models composed of hybrid methods. Ren et al. [26] proposed an integrated method named correntropy-induced loss-based sparse robust graph regularized extreme learning machine and applied it to the classification and recognition of cancer samples. Gao et al. [27] performed cancer classification based on SVM optimized by particle swarm optimization combined with artificial bee colony approaches, and the effectiveness of these methods was verified by the experimental results. In addition, with the continuous development of machine learning, many studies have shown that the application of ensemble learning to classification problems is often better than traditional classification algorithms and single classifiers, and it can also solve the problem of increased data volume and data diversification [23, 26]. Therefore, a large number of classification models based on ensemble learning have been proposed. For example, Lee et al. [5] developed an ensemble model based on random forest and deep neural network for cancer classification and achieved an accuracy of 94%. ALzubi et al. [28] used the boosted weighted optimization neural network ensemble classification algorithm to classify cancer patients, thereby improving the accuracy of cancer diagnosis. Ghiasi and Zendehboudi [29] proposed a classification algorithm based on random forest and extreme random tree of decision tree, which was applied to the classification of breast cancer, and verified the diagnostic performance of the algorithm. Li and Luo [30] proposed a performance-weighted voting model for cancer classification. This ensemble model was composed of five weak classifiers: logistic region, SVM, RF, XGBoost, and neural networks, which achieved high accuracy of tumor diagnosis.

Stacking is widely used as a more flexible combination classification model in ensemble learning. However, in the process of constructing the combination model, how to choose the base classifier and give full play to their effectiveness and how to choose the best secondary learner are problems worthy of attention. In addition, the types and characteristics of experimental data will also affect the effectiveness of the classification model. Therefore, in view of the above problems, first of all, we used the FCBF algorithm to reduce the data dimension and achieve the purpose of simplifying the classification model. In addition, four base classifiers (LIBSVM, KNN, C4.5, and RF) were used as the primary learners of the ensemble model. Meanwhile, cost-sensitive learning idea was introduced as a secondary learner to solve the imbalance of microarray gene expression data, so as to overcome these problems and achieve high-quality classification results.

## 3. Materials and Methods

### 3.1. Cancer Datasets

For evaluation of the effectiveness of the proposed method, we used nine groups of cancer datasets of two classes derived from the Kent Ridge Biomedical Dataset database. These datasets included central nervous system embryonal tumors (NervSys), leukemia, three groups of diffuse large B-cell lymphoma (DLBCL), prostate cancer, ovarian cancer, and two groups of lung cancer. A detailed description of these datasets is shown in Table 1.

Among these sample data, DLBCL1 was derived from Stanford data, including a total of 62 samples of two subtypes. DLBCL2 and DLBCL3 were selected from two sets of data detected by Harvard. DLBCL2 included two types of patients: those with DLBCL and those with follicular lymphoma. DLBCL3 comprised the outcome prediction data, including cured patient samples and relapsed patient samples. Lung cancer1 was derived from the University of Michigan, including ten normal samples and 86 diseased samples. Lung cancer2 contained 181 samples comprising 31 cases of malignant pleural mesothelioma and 150 cases of adenocarcinoma, with 12533 genes detected. Notably, the NervSys and DLBCL3 data were outcome prediction data, whereas the ovarian cancer data were protein data, and the remaining samples were from two categories of data.

### 3.2. Stacking Ensemble Learning Algorithm

Stacking, also known as stacked generalization [31], is a technology involving heterogeneous classifier collections. By integrating multiple different types of base classifiers and combining them into a strong classifier, the generalization ability of the strong classifier can be improved. The stacking ensemble learning algorithm adopted a two-layer framework structure, as shown in Figure 1. The main idea of this algorithm was to train the dataset with multiple primary learners first. Then, the prediction results obtained by each base classifier were used as the input of the metaclassifier to perform training again. Finally, the training result of the metaclassifier was the final prediction result. The stacking ensemble algorithm took into account the learning ability of the primary classifier and metaclassifier, so that the final classification performance was significantly improved [32–34].

### 3.3. KNN

KNN [35] is a classification algorithm in supervised learning and also a lazy learning algorithm. The algorithm has the advantages of simple use, rapid calculation, and good predictive effects. However, when the sample distribution is uneven, the prediction error also increases.

The basic idea of the algorithm was that if a prediction sample has *K*-nearest neighbors in the feature space, the category of the prediction sample was usually determined by most of the categories of the *K*-nearest neighbors. The effects and performance were optimized by selecting the *K* value, distance measurement method, and classification decision rules.

### 3.4. C4.5

The three commonly used decision tree algorithms [36] are Iterative Dichotomiser (ID3), C4.5, and CART. Among them, decision tree C4.5 was an improvement on ID3. The C4.5 algorithm used the information gain ratio as the index to select the best split, which accommodated continuous variables and missing values, thereby addressing the disadvantage of ID3's tendency to select attributes with many categories. Pruning could be performed during the construction of the tree to avoid overfitting.

### 3.5. RF

RF [37] is an ensemble algorithm that constructs a strong classifier by training multiple weak classifiers. The prediction results were determined by the average or voting of multiple base classifiers, thus giving the prediction model good accuracy and generalization ability. The decision tree was used as the base classifier in the RF. When making predictions, each decision tree in the forest participated in classification prediction. Finally, the classification with the highest number of votes was selected as the prediction value. The accuracy of RF depended on the strength of the base classifier and the dependence between them. Moreover, it was relatively robust to errors and outliers.

### 3.6. SVM

SVM [38] is a classic stability classifier. The SVM method was based on the VC dimension theory of statistical theory and the principle of minimum structural risk. The VC dimension represented the complexity of the problem. Normally, the higher the VC dimension, the more complex the function. SVM had advantages in handling nonlinear high-dimensional problems, and it is widely used in the classification and recognition fields [39].

For nonlinear samples, SVM used a kernel function to map the original data to a high-dimensional space, thus making the samples linearly separable. The optimal classification hyperplane was constructed to separate the samples correctly. Generally, different forms of kernel functions strongly affected the classification performance of SVM. Among them, the radial kernel function (RBF) [40] had fewer parameters and better performance and consequently was widely used in practical applications. The formula of the RBF kernel function can be expressed as follows:

(1) $$\begin{array}{c} K\left(x,x_{i}\right)=\exp\left(-\frac{{\left\|x-x_{i}\right\|}^{2}}{\sigma^{2}}\right), \end{array}$$

where *x* and *x*_*i*_ are two sample vectors, *K* is the value of the RBF kernel function, and *σ* is a free parameter.

### 3.7. CSNB

Cancer gene expression data are a type of unbalanced data [41]. Traditional classification algorithms often do not consider the factor of misclassification cost, thereby leading to classification results that tend to focus on the learning of large categories while ignoring the learning of small categories. In this experiment, the idea of cost sensitivity was introduced into a naive Bayes classification algorithm to make it sensitive to cost. In this way, the recognition rate of rare classes was improved, and the validity of classification was strengthened.

First, the definition of misclassification cost was given. Taking a binary classification dataset as an example, let the *c*_0_ class be the minority class and the *c*_1_ class be the majority class. The misclassification cost can usually be represented by a 2 × 2 cost matrix, and each element in the matrix represents the misclassification cost of samples [42].

(2) $$\begin{array}{c} C=\left[\begin{array}{cc} C_{00} & C_{01}\\ C_{10} & C_{11} \end{array}\right], \end{array}$$

where *C*_*ij*_ represents the cost of mistakenly classifying samples that are *i* classes into *j* classes. Generally, for the rationality condition of two classification problems [43], correct classification is not considered to bring losses; consequently, the cost of misclassification is 0. However, the cost of small classes being misclassified into large classes is much higher than that of large classes being misclassified into small classes. Therefore, we can derive the following relationship: *C*_00_ = *C*_11_ = 0 and *C*_01_ > *C*_10_.

After the cost matrix is determined, the naive Bayes theory is used to construct the risk function [38]. When a sample *x* with an unknown category is classified by a classification algorithm, the sample *x* can be represented by a vector (*a*_1_, *a*_2_, *a*_3_,⋯, *a*_*n*_). The probability that it belongs to the category *c*_*j*_ is *P*(*c*_*j*_ |  *x*), which is expressed by the Bayesian formula as

(3) $$\begin{array}{c} P\left({\text{c}}_{j}\;|\;x\right)=\frac{P\left(x\;|\;c_{j}\right)P\left(c_{j}\right)}{P\left(x\right)}=\frac{P\left(a_{1},a_{2},a_{3},\cdots a_{n}\;|\;c_{j}\right)P\left(c_{j}\right)}{P\left(x\right)}. \end{array}$$

When its category is determined to be *c*_*j*_, the expected misclassification cost is

(4) $$\begin{array}{c} R\left(c_{j}\;|\;x\right)=\underset{i}{\sum }P\left(c_{i}\;|\;x\right)C_{ij}, \end{array}$$

where *P*(*c*_*i*_ |  *x*) represents the posterior probability that sample *x* belongs to the *c*_*i*_ category. Its value is obtained by the naive Bayes formula. Furthermore, the corresponding categories are determined by minimizing the posterior probability as follows:

(5) $$\begin{array}{c} c=\underset{j=0,1}{\arg\min}\left\{R\left(c_{j}\left|x\right.\right)\right\}. \end{array}$$

The sample *x* is finally predicted to be a certain category *c*_*j*_ that makes *R*(*c*_*j*_  |  *x*) have a minimum value, which can be expressed as

(6) $$\begin{array}{c} R\left(c_{j*}\;|\;x\right)=\min_{j}R\left(c_{j}\;|\;x\right), \end{array}$$

where formula (6) is the CSNB formula.

### 3.8. FCBF

FCBF [39] is a supervised fast filtering feature selection algorithm. Its core idea is to define *C*-correlation and *F*-correlation, where *C*-correlation is the degree of correlation between features and categories and *F*-correlation is the degree of correlation between features. When a feature has high *C*-correlation with a category and low *F*-correlation with other selected features, the feature is marked as an important feature. In this algorithm, symmetric uncertainty (SU) was adopted as the standard to measure the degree of correlation. SU is defined as the standardized information gain:

(7) $$\begin{array}{c} \text{SU}\left(X,Y\right)=2\left[\frac{\text{IG}\left(X\left|Y\right.\right)}{H\left(X\right)+H\left(Y\right)}\right], \end{array}$$

where *X* and *Y* represent two random variables, IG(*X* | *Y*) denotes the information gain, and *H*(*X*) represents the information entropy.

### 3.9. The Proposed CSNB Stacking Algorithm

In this article, the FCBF algorithm was first used to reduce the dimensionality of the datasets. Then, LIBSVM, KNN, C4.5, and RF were used as primary learners. In addition, given the unbalanced classification of cancer gene expression data, the naive Bayes with embedded cost sensitivity was adopted as the metalearner of the stacking ensemble. In the experiment, the 5 × 10-fold nested cross-validation method was used to divide the data to prevent overfitting. The experimental process is shown in Figure 2.

## 4. Results

### 4.1. Feature Selection

Cancer datasets contain many genes that are irrelevant and redundant for classification, thus leading to more complex classification tasks and inaccurate classification results. In fact, few informative genes are known to directly affect the classification results. Therefore, to save time and calculation costs and obtain better classification performance, we used the FCBF method to quickly and effectively reduce the dimensionality of the cancer datasets before classification, by discarding features making little or no contribution to classification. In this article, data were preprocessed first, and FCBF was used in WEKA for feature selection. The data information after reduction is provided in Table 2.

As shown in Table 2, the feature dimensions of the nine cancer datasets were greatly reduced after feature selection with the FCBF algorithm. Among them, ovarian cancer was reduced from the original 15154 attributes to 30, whereas the number of features of DLBCL2 was decreased from 7129 to 27. In addition, lung cancer ultimately retained only one important feature among 7129 original features. Hence, after the feature reduction by the FCBF algorithm, the subsequent classification task was greatly simplified.

### 4.2. Cancer Classification

In this article, the nine cancer datasets after feature reduction are used as the input to the proposed method CSNB stacking classifier for classification. To test the quality of the proposed method, we compared this method with CSKNN stacking, CSC4.5 stacking, CSLIBSVM stacking, bagging, AdaBoost, CSNB, NB, LIBSVM, KNN, RF, andC4.5.

Among these methods, the primary learners with the CSKNN stacking, CSC4.5 stacking, and CSLIBSVM stacking were the same as with the proposed method, but the metalearners were different. CSKNN stacking adopts embedded cost-sensitive KNN as a metalearner for combinatorial learning. CSC4.5 stacking used embedded cost-sensitive C4.5 as a metalearner for classification, whereas the metalearner of CSLIBSVM stacking applies embedded cost-sensitive LIBSVM. Both bagging and AdaBoost ensemble methods used CSNB as the base classifier. The CSNB algorithm introduced cost-sensitive information into naive Bayes, thus making it sensitive to cost and emphasizing the learning of small samples. The above classification models all used cost-sensitive learning. In addition, several other comparison methods exist. Among them, the naive Bayes algorithm was simple and provided stable classification efficiency, but it was highly sensitive to the expression form of the input data; for example, if the training data error is large, the predictive effect will be poor. The LIBSVM classification algorithm had few parameters, flexible operation, and broad application capability. KNN was simple and effective and had low training costs, but it was computationally expensive. RF adopted an integrated algorithm with high accuracy and fast training speed, but the training required large amounts of time and space. Moreover, the RF model was prone to overfitting for sample sets with high noise. The classification rules generated by the C4.5 algorithm were easy to understand and have high accuracy; this algorithm handled discrete and continuous data, but its computational efficiency was low.

Furthermore, owing to the small training set, we evaluated the classification performance with 5 × 10-fold nested cross-validation to avoid overfitting. That is, the data were first divided by the 5-fold cross-validation method, and then, the datasets were divided according to the 10-fold cross-validation method before the primary classifier of stacking carries out the training data. The classification accuracy, recall rate, *F*-score, specificity, and receiver operating characteristic (ROC) curves were used to evaluate the effectiveness of the proposed method. The final classification accuracy results are shown in Table 3.

As shown in Table 3, the first row represented the classification results of the proposed CSNB stacking method, which always obtained the best value for the nine datasets. In these classification results, such as those with NervSys, the proposed CSNB stacking method achieved the same accuracy as CSC4.5 stacking (both 90%, a value higher than those of other methods). For the DLBCL3 and prostate cancer datasets, the method proposed in this article, compared with other classification methods, had the highest classification accuracy. In addition, the proposed classification model achieved 100% classification accuracy on the leukemia, DLBCL1, ovarian cancer, and lung cancer2 datasets. According to the classification results, the classification method based on a stacking ensemble was better than the single classification model. To visually demonstrate the classification effect of different models, we have converted the experimental results in Table 3 to a line graph, as shown in Figures 3 and 4. Because the classification results for the leukemia, DLBCL1, and ovarian datasets were all 100%, they were not shown in the figure. In Figure 4, the remaining classification methods were combined and compared with the proposed method. Similarly, because lung1 achieved 98% in these comparison methods, it was also not shown in the figure.

Figure 5 shows the values of the recall rates obtained by the various classification methods on nine cancer datasets. The results show that the proposed CSNB stacking method achieves the highest recall rate on all nine datasets, followed by the CSKNN stacking method. For DLBCL3 and prostate cancer, the recall rate of the proposed method reached 87.90% and 95.10%, respectively; these results were superior to those of other classification models.

Figures 6 and 7 illustrate the specificity values obtained by the various classification methods on nine cancer datasets.  Figure 6 shows the comparison between the proposed method and the other five ensemble classifiers. Since the specificities of the six ensemble classifiers in the three datasets of leukemia, DLBCL1, and ovarian cancer were all 1, they were not shown in the figure.  Figure 7 is a comparison of other remaining classification models and the proposed method. It can be seen from the figure that the proposed methods in this paper can obtain better specificity on nine datasets. In addition, compared with other ensemble classifiers, the proposed method had a better classification effect and achieves specificity of 0.9 and 1 on lung1 and lung2 datasets, respectively. However, CSC4.5 stacking performed poorly, especially for the lung1 dataset, with a specificity value of 0. Although C4.5 achieved a specificity of 1 on the lung1 dataset, the results on the remaining eight datasets were not good.

Table 4 lists the *F*-score of different classification methods on each cancer dataset. As can be seen from the table, the proposed method obtained the highest *F*-score on all nine datasets. Since the *F*-score represents the harmonic mean value of precision and recall rate, the experimental results further verified the effectiveness of the proposed method.

In order to display the ROC curves of different classification models more clearly and intuitively, we selected NervSys and prostate datasets from nine datasets for graphing. In addition, we divided all classifiers into two groups to show them more aesthetically and clearly.  Figure 8 shows the ROC curves of the NervSys dataset on different classifiers.  Figure 9 shows the ROC curves of the prostate dataset on different classifiers. It can be seen from the figure that the proposed classification model in this study had a better performance, and the curve corresponding to CSNB stacking was closer to the upper left corner of the ROC chart, which further proved the great advantage of the proposed method in dealing with cancer datasets.

## 5. Discussion

As a combinatorial learning method, the stacking method is supported by less theoretical research than the boosting and bagging combination method, but it is welcomed by many researchers because of its strong flexibility and scalability in algorithms [44, 45]. However, the choice of the output data type of the base learner and the metalearner are longstanding problems in the stacking method. Some researchers favor using the output probability of the base learner as the input of the secondary learner. In addition, if some relatively simple learners are selected as primary learners and more complex learners are selected as metalearners, the stacking performance will be more robust in terms of classification accuracy [46, 47]. Therefore, herein, we propose the novel combination classification model CSNB stacking and perform experimental verification.

The datasets selected in this experiment were diverse, including prognostic data, protein data, and two-category data. The experimental results showed that the proposed method achieved the best classification accuracy in different types of cancer datasets, thus reflecting the superiority of the CSNB stacking classification model in processing cancer datasets. On the other hand, through the experimental verification, the four base classifiers selected in this study constitute the primary learner of stacking, which is a satisfactory combination. At the same time, the cost-sensitive idea was introduced into the metalearner of stacking, which can well deal with the problem of unbalanced data. In addition, the proposed classification combination model was superior to the single classifier and ensemble algorithm in terms of stability and generalization ability, and it achieved better classification results. Furthermore, the proposed method provided a feasible reference scheme for the two-classification problem, and it may potentially aid in cancer prediction, identification, and classification.

## 6. Conclusion

Owing to its high incidence and mortality, cancer has always been a threat to human health. Its complexity and variability make clinical diagnosis and treatment difficult. The emergence of cancer gene expression profiles, by synchronously tracking the expression levels of many genes, is important for early diagnosis of cancer at the molecular level. However, the analysis and processing of gene expression data are accompanied by problems such as high dimensionality, relatively small samples, high noise, and class imbalance. Therefore, to improve the quality of cancer classification and determine the genes that contribute to classification, we proposed a novel method for gene expression data classification: CSNB stacking, based on a CSNB stacking ensemble. This algorithm is based on the traditional stacking algorithm. In addition, because of the imbalanced characteristics of cancer gene expression data, we adopted the embedding CSNB as the metalearner of the stacking ensemble.

In the experiment, FCBF was first used to reduce the dimensionality of the data and discarded the irrelevant and redundant attributes. Then, the feature subset was input into the CSNB stacking classification model for classification. The experimental results for nine sets of cancer datasets demonstrated that the CSNB stacking method achieved the best classification performance among the tested methods. Simultaneously, this method had advantages in processing outcome prediction data, protein data, and two categories of data, and it therefore should have high guidance potential and clinical value for cancer classification and prognosis prediction.

In addition, through the comparison and analysis of the experimental results, the superiority of the proposed method in the binary classification problem was verified. Our next step will be to expand to the multiclassification task on the basis of the algorithm, to explore its effectiveness. Simultaneously, to make the algorithm more conducive to solving practical problems, we will also focus on combining multiple types of data to achieve more detailed analysis in the future.

## Figures and Tables

**Figure 1:** Ensemble learning method based on stacking.

**Figure 2:** The experimental flow of the proposed method.

**Figure 3:** Cancer classification accuracy of different ensemble methods.

**Figure 4:** Cancer classification accuracy of different methods.

**Figure 5:** Recall rate of different methods.

**Figure 6:** Specificity of different ensemble methods.

**Figure 7:** Specificity of different methods.

**Figure 8:** ROC curves of NervSys by different classification methods.

**Figure 9:** ROC curves of the prostate dataset by different classification methods.

**Table 1:** Details of cancer datasets.

Datasets	Samples	No. of genes	Classes	Labels
NervSys	60	7129	2	Outcome prediction
Leukemia	72	7129	2	Two categories
DLBCL1	47	4026	2	Two categories
DLBCL2	77	7129	2	Two categories
DLBCL3	58	7129	2	Outcome prediction
Prostate	102	12600	2	Cancer or not
Ovarian	253	15154	2	Protein data
Lung1	96	7129	2	Cancer or not
Lung2	181	12533	2	Two categories

**Table 2:** Reduced attributes by FCBF.

Datasets	Original attributes	Reduced attributes
NervSys	7129	28
Leukemia	7129	51
DLBCL1	4026	60
DLBCL2	7129	73
DLBCL3	7129	27
Prostate	12600	77
Ovarian	15154	30
Lung1	7129	1
Lung2	12533	128

**Table 3:** Classification accuracy (%) of different methods.

Datasets	NervSys	Leukemia	DLBCL1	DLBCL2	DLBCL3	Prostate	Ovarian	Lung1	Lung2
CSNB stacking	90.00	100	100	98.70	87.93	95.10	100	98.96	100
CSKNN stacking	83.33	100	100	98.70	84.48	92.16	100	98.96	100
CSC4.5 stacking	90.00	100	100	98.70	86.21	93.14	100	89.58	99.45
CSLIBSVM stacking	86.67	100	100	97.40	77.59	92.16	100	92.71	99.45
Bagging	83.33	100	100	97.40	84.48	93.14	100	98.96	100
AdaBoost	81.67	100	100	96.10	84.48	95.10	100	98.96	100
CSNB	76.67	100	100	96.10	86.21	92.16	100	98.96	100
NB	76.67	100	100	96.10	86.21	92.16	100	98.96	100
LIBSVM	86.67	100	100	98.70	82.76	94.12	100	98.96	99.45
KNN	86.67	100	95.74	93.51	70.69	89.22	100	98.96	100
RF	88.33	98.61	100	96.10	86.21	94.12	99.60	98.96	99.45
C4.5	75.00	81.94	78.72	84.42	72.41	88.24	98.02	98.96	95.58

**Table 4:** *F*-score of different classification methods.

Datasets	NervSys	Leukemia	DLBCL1	DLBCL2	DLBCL3	Prostate	Ovarian	Lung1	Lung2
CSNB stacking	0.900	1.00	1.00	0.987	0.878	0.951	1.00	0.989	1.00
CSKNN stacking	0.829	1.00	1.00	0.987	0.844	0.922	1.00	0.989	1.00
CSC4.5 stacking	0.899	1.00	1.00	0.987	0.861	0.931	1.00	0.945	0.995
CSLIBSVM stacking	0.869	1.00	1.00	0.974	0.775	0.922	1.00	0.909	0.995
Bagging	0.829	1.00	1.00	0.974	0.842	0.931	1.00	0.989	1.00
AdaBoost	0.813	1.00	1.00	0.961	0.844	0.951	1.00	0.989	1.00
CSNB	0.767	1.00	1.00	0.961	0.862	0.922	1.00	0.989	1.00
NB	0.767	1.00	1.00	0.961	0.862	0.922	1.00	0.989	1.00
LIBSVM	0.867	1.00	1.00	0.987	0.821	0.941	1.00	0.989	0.995
KNN	0.869	1.00	0.957	0.937	0.707	0.892	1.00	0.989	1.00
RF	0.879	0.986	1.00	0.960	0.860	0.941	0.996	0.989	0.994
C4.5	0.741	0.822	0.785	0.838	0.724	0.882	0.980	0.952	0.955

## Data Availability

The data used to support the findings of this study are available from the corresponding author upon request.
